# The Coral Reefs Optimization Algorithm: A Novel Metaheuristic for Efficiently Solving Optimization Problems

**DOI:** 10.1155/2014/739768

**Published:** 2014-07-22

**Authors:** S. Salcedo-Sanz, J. Del Ser, I. Landa-Torres, S. Gil-López, J. A. Portilla-Figueras

**Affiliations:** ^1^Department of Signal Theory and Communications, Universidad de Alcalá, Escuela Politécnica Superior, 28871 Alcalá de Henares, Spain; ^2^Tecnalia Research & Innovation., Parque Tecnológico de Bizkaia, Zamudio, 48170 Bizkaia, Spain

## Abstract

This paper presents a novel bioinspired algorithm to tackle complex optimization problems: the coral reefs optimization (CRO) algorithm. The CRO algorithm artificially simulates a coral reef, where different corals (namely, solutions to the optimization problem considered) grow and reproduce in coral colonies, fighting by choking out other corals for space in the reef. This fight for space, along with the specific characteristics of the corals' reproduction, produces a robust metaheuristic algorithm shown to be powerful for solving hard optimization problems. In this research the CRO algorithm is tested in several continuous and discrete benchmark problems, as well as in practical application scenarios (i.e., optimum mobile network deployment and off-shore wind farm design). The obtained results confirm the excellent performance of the proposed algorithm and open line of research for further application of the algorithm to real-world problems.

## 1. Introduction

In the last years, huge research efforts have been conducted towards solving hard optimization problems, by well balancing the trade-off between the complexity incurred by the utilized method and the optimality of the produced solutions. These problems, often characterized by search spaces of high dimensionality (either discrete or continuous), nonlinear objective functions and/or stringent constraints arise frequently in science and engineering applications. In such fields, classical optimization approaches do not provide in general good solutions to these problems or are just not applicable, due to the unmanageable search space structure or its huge size.

In this context, modern optimization heuristics and metaheuristics have been lately the core of research, aimed at solving the aforementioned lack of efficient methods. A good number of such algorithms are* bioinspired* techniques such as evolutionary algorithms (EA), which includes a whole family of techniques such as genetic algorithms [1], evolutionary strategies [2], evolutionary programming [3], and differential evolution [4]. These schemes are based on concepts borrow from natural evolution and survival of the fittest individuals in nature. Likewise, ant colonies optimization (ACO) [5] is based on the social behavior of ants, whereas artificial immune system (AIS) algorithms [6] focus on imitating the behavior of the immune system in animals. In this same line of research, particle swarm optimization (PSO) approaches [7] are in essence elegant algorithms specially well-suited for continuous optimization problems. They imitate the behavior of birds flocks or fish schools. There have been more research activity on bioinspired metaheuristics, with approaches such as artificial bee colony [8], which imitates the bees behavior when locating and bring food to the hive, as well as other recently proposed techniques such as the gravitational search algorithm (GSA), [9], inspired by the law of the gravity, the invasive weed optimization algorithm (IWO), [10], based on weed growth and their invasive properties, the hunting search (HS), [11], based on how group of animals hunt, the biogeography-based optimization algorithm (BBO), [12, 13], based on the geographical distribution of living organisms, optimization based on virus infection [14], and on colonies of bacteria [15, 16], the bat algorithm [17, 18], based on the behaviour of bats and its capability for echolocation of objects, the amoeba algorithm [19] that uses the intelligence of groups of amoebas to explore solutions to complicated problems in networks, the collide bodies optimization algorithm [20], based on the behaviour of bodies colliding at different speeds, the ray optimization algorithm [21], based on particles that follow the snell's law for ray of light, or the so-called cuckoo search approach [22], built upon the reproduction and breeding of the cuckoo bird.

There exist other metaheuristic optimization approaches not straightforwardly classifiable as bioinspired approaches; instead, they are based on alternative concepts or processes that make them worth to be considered in this literature review. For instance, simulated annealing [23] (SA) is a well-known metaheuristic based on the process of annealing in metallic materials. It consists of heating a substance and then cooling it down slowly, until a final strong molecular structure is obtained. This process can be artificially simulated in order to solve optimization problems. There are several variants of this algorithm such as simulated quenching [24]. Another recently proposed metaheuristic is the harmony search (HS) algorithm [25], which has been successfully applied to numerous optimization problems in the last few years. HS is inspired by the improvisation process of musicians, that is, the process by which the musicians (who may have never played together before) refine, through variation and check, their individually improvised notes, resulting in an aesthetic harmony, played by the entirety of musicians in the orchestra. Other modern heuristics recently proposed for optimization problems include, among others, the teaching-learning-based optimization (TLB) [26], based on the process of teaching-learning produced by different teachers in a class of students; the society and civilization algorithm (SaC) [27], which simulates the social behavior of humans; the imperialist competitive algorithm (ICA) [28], which makes optimization based on imperial-colonies competition; the artificial chemical reaction optimization algorithm (ACROA) [29], based on different types of chemical reactions (synthesis, decomposition, redox, etc.); or the electromagnetic-like algorithm [30, 31], based on physics of electrically charged particles, repelling and attracting each other in a multidimensional space.

In this paper we present a novel bioinspired metaheuristic for optimization problems, which will be hereafter coined as the coral reefs optimization (CRO) algorithm. The CRO algorithm is based on an artificial simulation of the process of coral reefs' formation and reproduction. During this process, the CRO algorithm emulates different phases of coral reproduction and fight for space in the reef, which ultimately renders an efficient algorithm for solving difficult optimization problems. The proposed CRO approach can be regarded as a cellular-type evolutionary scheme [32], with superior exploration-exploitation properties thanks to the particularities of the emulated reef structure and coral reproduction. The performance of the proposed approach has been tested in different benchmark problems and in two different practical applications (namely, mobile network deployment and wind farm design), obtaining very good results in comparison with alternative approaches in the literature.

The rest of this paper is structured as follows. For the sake of self-completeness of the paper, the next section provides an introduction to coral reefs and corals' structure and reproduction. Next, Section 3 presents the CRO algorithm in detail, including an analysis of similarities and differences with other existing metaheuristics.  Section 4 shows the performance of the CRO algorithm in different optimization problems. Finally, Section 5 ends the paper by giving some concluding remarks.

## 2. Corals and Coral Reefs

This section describes some important properties of corals and coral reefs that will be simulated by our CRO approach. We first describe some characteristics of corals and reefs, and then we focus on corals reproduction.

### 2.1. Corals and Reef Formation

A coral is an invertebrate animal belonging to the group phylum: Cnidaria, which also includes sea anemones, hydras, or jellyfishes [33]. In fact, a more detailed classification includes corals in the* Anthozoa* class, together with sea anemones, sea pens, or sea pansies. These animals are characterized by their ability to subsist either as individuals or in colonies of polyps, living attached to a substrate. There are more than 2500 different species of corals, living in shallow and deep waters, and each year new species are found and described.

An important subclass of corals are reef-building corals, also known as* hermatypic* or simply* hard corals*. Hard corals are usually shallow-water animals that produce a rigid skeleton of calcium carbonate, segregated from their base. A coral reef is formed by hundred of hard corals, cemented together by the calcium carbonate they produce. Periodically, the polyp lifts off its basal plate of calcium carbonate and secrete a new one, forming a tiny chamber that will contribute to the coral's skeleton. Polyps continuously build these chambers in the reef, so finally the complete reef grows upwards. Living corals grow on top of the skeletons of calcium carbonate of their dead predecessors. A coral reef is usually formed by corals living in colonies or on its own. A colony is composed of a single specie of coral, but a reef's structure can comprise multiple types of species. In fact, a coral reef finally ends up as a truly ecosystem, in which a diverse collection of animals and plants interact with each other, as well as with their environment. In addition to corals, many other animals and plants live in and from the reef, such as algae, sponges, sea anemones, bryozoans, sea stars, crustaceans (e.g., shrimps, crabs, lobsters), octopuses, squids, clams, snails, and other mollusca. And, of course, a huge variety of fish that find shelter and food in the reef.

In general, hard coral species require free space to settle and grow. Although a priori the implementation of this settlement procedure might be easy for a potential new member of the reef, in practice free space is an extremely limited resource in the reef environment [34]. As a result, species often compete with each other or exhibit aggressive behavior to secure or maintain a given plot of substrate [35]. Different strategies used by corals to compete for the space have been thoroughly described in the literature [35, 36]. Among them, fast growing is deemed as the most used and simple strategy since it grounds on the fact that there are corals that have evolved to yield a faster growth rate than others. When a fast-growing coral sets near a slow-growing one, the former attacks the latter by overtopping it. The underlying coral suffers from light deficiency, thus affecting its ability to conduct photosynthesis and to get into contact with food particles. As time evolves, overtopping by fast-growing species kills the slower-growing species underneath. Other aggressive strategies carried out by some species of corals include sweeper tentacles (i.e., detect and damage adjacent coral colonies),* mesenterial* filaments (namely, enabling external digestion of neighboring colonies), and* terpenoid compounds* (coral chemical warfare).

### 2.2. Coral Reproduction

Corals can reproduce in two different modes: sexual or asexual. In fact, an individual polyp may use both modes within its life time [33]. Furthermore, sexual reproduction can be either external or internal, depending on the coral species.

#### 2.2.1. Sexual External Reproduction: Broadcast Spawning

The majority of hard corals species resort to a sexual external reproduction method known as* broadcast spawning* [37]: every coral produces male and/or female (some species of corals are hermaphrodites) gametes that are massively released out to the water.  Figure 1 shows a recreation of a coral spawning event in a reef. Once the egg and sperm meet together, a larva (also called* planula*) is produced. Planulae float in the water until they find a proper space to attach and start growing a polyp [38]. In the majority of reefs, the phenomenon of coral spawning occurs as a synchronized event. This timing is crucial for successful reproduction, since corals can not move to force reproductive encounters. There are different natural aspects that affect the timing of the corals' spawning, such as temperature, day length, or temperature change rate.

#### 2.2.2. Sexual Internal Reproduction: Brooding

Brooding is a method of internal reproduction used by some species of corals. In this reproduction mode, some female polyps contain eggs that are not released to the water. Instead, sperm released by other male corals of the same species gets inside the polyp and fertilizes the eggs, producing small planulae. These planulae are released later through the mouth of the coral in an advanced stage of development, so it becomes easier for these planulae to set onto hard substrate without being attacked or depredated. There has also been described a type of brooding reproduction in hermaphrodite corals [39].

#### 2.2.3. Asexual Reproduction: Budding or Fragmentation

Budding is a form of asexual reproduction in corals: basically, new polyps bud off from parent polyps to expand or begin new coral colonies [40]. Budding occurs when the coral has grown enough to produce budding. Fragmentation is a process similar to budding, but it is caused by external phenomena (e.g., storms or boats' grounding), and usually a larger part of the coral is divided in comparison to budding [41]. As such, in fragmentation a part of a coral colony is separated from the parent polyps. Individuals broken off this way from the main colony are able to keep growing and finally establishing a new colony far way from the parent one if conditions are favorable. It is important to note that both budding and fragmentation processes produce polyps that are genetically identical to the parent polyp/colony.

### 2.3. Reef Longevity and Causes of Death

There are not reliable statistics on corals' lifespan. However, it is well known that coral colonies can live for several centuries. Corals and coral reefs must face different hazards during their life. In larva state, corals are massively depredated by fishes and other predators. However, the huge number of larvae produced in broadcast spawning reproduction ensures that enough polyps settle in favorable ground and start forming a colony. On the other hand, coral polyps encounter many types of predators including sea stars, parrot-fishes, or butterfly-fishes. Human activities (e.g., fishing activities or industrial processes that increase ocean pollution) and climate changes (increase of the oceans' temperature, among others) also contribute to the loss of living corals [42].

## 3. The Coral Reefs Optimization Algorithm

Having these fundamentals on the corals' reproduction and formation in mind, the CRO algorithm tackles optimization problems by modeling and simulating all the distinct processes explained in Section 2. Let Λ be a model of reef, consisting of a *N* × *M* square grid. We assume that each square (*i*, *j*) of Λ is able to allocate a coral (or colony of corals) Ξ_*i*,*j*_, representing different solutions to our problem, encoded as strings of numbers in a given alphabet *I*. The CRO algorithm is first initialized at random by assigning some squares in Λ to be occupied by corals (i.e., solutions to the problem) and some other squares in the grid to be empty; that is, holes in the reef where new corals can freely settle and grow. The rate between free/occupied squares in Λ at the beginning of the algorithm is an important parameter of the CRO algorithm, which will be denoted in what follows as 0 < *ρ*_0_ < 1.  Figure 2(a) exemplifies this reef model using a 5 × 6 grid, whereas Figure 2(b) illustrates an initialization of the reef with corals and coral colonies representing solutions to a given problem. Note that in this example *ρ*_0_ = 9/21 ≈ 0.43. Each coral is labeled with an associated* health* function *f*(Ξ_*ij*_) : *I* → *R* that represents the problem's objective function. Note that the reef will progress as long as healthier (stronger) corals (which represent better solutions to the problem at hand) survive, while less healthy corals perish.

After the reef initialization described above, a second phase of reef formation is carried out by the CRO algorithm. To this end, a simulation of the corals' reproduction in the reef is done by sequentially applying different operators. This sequential set of operators is then applied iteratively until a given stop criteria is met. Thus, we define different operators for modeling sexual reproduction (broadcast spawning and brooding), asexual reproduction (budding), and polyps depredation. In both sexual and asexual reproduction we give the conditions under which new corals effectively get attached to the reef or are depredated while at the larvae phase, it is as follows:

(*1) Broadcast Spawning (External Sexual Reproduction).* The modeling of coral reproduction by* broadcast spawning* consists of the following steps.

(1a) In a given step *k* of the reef formation phase, select uniformly at random a fraction of the existing corals *ρ*_*k*_ in the reef to be broadcast spawners. The fraction of broadcast spawners with respect to the overall amount of existing corals in the reef will be denoted as *F*_*b*_. Corals that are not selected to be broadcast spawners (i.e., 1 − *F*_*b*_) will reproduce by brooding later on, in the algorithm.
(1b) Select couples out of the pool of broadcast spawner corals in step *k*. Each of such couples will form a coral larva by sexual crossover, which is then released out to the water. Note that, once two corals have been selected to be the parents of a larva, they are not chosen anymore in step *k* (i.e., two corals are parents only once in a given step). These couple selection can be done uniformly at random or by resorting to any fitness proportionate selection approach (e.g., roulette wheel).

(*2) Brooding (Internal Sexual Reproduction).* As previously mentioned, at each step *k* of the reef formation phase in the CRO algorithm, the fraction of corals that will reproduce by brooding is 1 − *F*_*b*_. The brooding modeling consists of the formation of a coral larva by means of a random mutation of the brooding-reproductive coral (self-fertilization considering hermaphrodite corals). The produced larva is then released out to the water in a similar fashion than that of the larvae generated in step (1b).

*(3) Larvae Setting.* Once all the larvae are formed at step *k* either through broadcast spawning (1) or by brooding (2), they will try to set and grow in the reef. First, the health function of each coral larva is computed. Second, each larva will randomly try to set in a square (*i*, *j*) of the reef. If the square is empty (free space in the reef), the coral grows therein no matter the value of its health function. By contrast, if a coral is already occupying the square at hand, the new larva will set only if its health function is better than that of the existing coral. We define a number *κ* of attempts for a larva to set in the reef: after *κ* unsuccessful tries, it will be depredated by animals in the reef.

*(4) Asexual Reproduction.* In the modeling of asexual reproduction (budding or fragmentation), the overall set of existing corals in the reef are sorted as a function of their level of healthiness (given by *f*(Ξ_*ij*_)), from which a fraction *F*_*a*_ duplicates itself and tries to settle in a different part of the reef by following the setting process described in Step (3).

*(5) Depredation in Polyp Phase.* Corals may die during the reef formation phase of the CRO algorithm. At the end of each reproduction step *k*, a small number of corals in the reef can be depredated, thus liberating space in the reef for next coral generation. The depredation operator is applied with a very small probability *P*_*d*_ at each step *k*, and exclusively to a fraction *F*_*d*_ of the worse health corals in Λ. For the sake of simplicity in the parameter setting of the CRO algorithm, the value of this fraction may be set to *F*_*d*_ = *F*_*a*_. Any other assignment may also apply provided that *F*_*d*_ + *F*_*a*_ ≤ 1 (i.e., no overlap between the asexually reproduced and the depredated coral sets).

Figure 3 illustrates the flow diagram of the CRO algorithm referencing the two CRO phases (reef initialization and reef formation), along with all the operators described above.

### 3.1. Analysis of the CRO Algorithm

The CRO algorithm differs from other existing bioinspired algorithms in several peculiarities. In this subsection we analyze the structure of the CRO, similarities, and differences with other metaheuristics. An insight on the proper choice of the CRO parameters is also provided.

We have already stated that the CRO structure resembles that of a cellular evolutionary algorithm [32]. This implies that it can be programmed as a fully parallel algorithm in a cluster of microprocessors. Of course, the implementation in a single processor is possible, and in fact it is expected to be the most widely implemented method. However, a major difference with cellular genetic and evolutionary algorithms is that in the CRO approach there are not neighborhoods defined in the grid. Instead, the CRO implements different processes based on corals reproduction and coral reef formation. In cellular evolutionary algorithms, the definition of neighborhoods in the grid is the key ingredient for the good performance of the algorithm, since a diffusion of solutions among the different neighborhoods in the grid is performed [32]. On the contrary, the CRO performance is driven by the fight for the space in the reef; that is, the fundamental point is the presence of holes in the reef that grant poorer solutions a possibility to survive. Note that the algorithm should be a priori structured in such a way that at the first stages this probability of survival of poor solutions is high (to favor the explorative capabilities of the search process), whereas in the last stages it should be made almost negligible (correspondingly, to make the algorithm exploit promising potential solutions detected during the evolutionary process). In the CRO, this tradeoff is controlled by two parameters: (1) in the reef formation, by the initial rate between free/occupied squares *ρ*_0_, and (2) in the last stages of the algorithm, by the depredation probability *P*_*d*_, which controls the appearance of available space in the reef when *ρ*_*k*_ gets close to 1.

Regarding the exploration/explotaition capabilities of the algorithm, it is interesting to observe that the CRO adopts concepts from evolutionary computation and simulated annealing algorithms, but with new variants. The exploration phase of the algorithm is carried out by operators that simulate the sexual and asexual reproductive processes of corals. The major exploration structure is the broadcast spawning process which should be carried out with a high probability, whereas the brooding reproduction is important for avoiding local optima. The budding (asexual reproduction) ensures that the best solutions replicate and span over the reef, so this process contributes to the exploitation phase of the CRO algorithm. As mentioned before, the fight for space in the reef is crucial in this exploitation phase. In this context, it is important to highlight that the exploitation phase resulting from the CRO is quite similar to the obtained by means of a simulated annealing algorithm, where the temperature of the system controls this phase, and the cooling rate is the key factor. In the CRO approach, the free/occupied rate is the factor that controls this exploitation phase.

We could also establish a first analysis of the parameters values of the CRO in terms of its intuitive theoretical behavior. Note, however, that the optimal specific values will be different in each case, so a sensitivity analysis of the CRO parameters must be carried out before its application to new problems. The initial free/occupied squares (*ρ*_*o*_) should be enough to allow new poorer solutions to have enough survival probabilities. Thus, a value for *ρ*_*o*_≃0.4 may be reasonable. On the other hand, it is intuitive that in the first steps of the algorithm the depredation probability *P*_*d*_ should be null, whereas in the final steps of the CRO, with the reef potentially complete with corals, a small value of this probability could help to avoid getting stuck in suboptimal solutions. Thus, a value of *P*_*d*_ in the interval [0,0.1] could be suitable for most applications, for example, if the stopping criteria is a maximum number of iterations, by imposing a linear progression of *P*_*d*_ with 0 as initial value and 0.1 at the end of the algorithm. Other parameters to be studied are the fractions *F*_*b*_ and *F*_*a*_ associated with coral reproduction. A high value of corals applying broadcast spawning is needed in order to ensure an efficient exploration of the search space. On the other hand, a small value of brooding and asexual reproduction is advisable. Therefore *F*_*b*_≃0.9 and *F*_*a*_≃0.1 could be a good starting parameter set.

Finally, a note on the computational complexity of the CRO is needed to close this analysis. In order to do this, we consider a situation where we establish a number of function evaluations for a given optimization problem. If this is the case, the computational cost of the algorithm will depend on the different operators applied to guide the search and exploit the solutions found. We can use a well-known algorithm for comparison purposes such as an evolutionary algorithm (EA). A basic EA with the same number of function evaluation implements operators of crossover, mutation, and selection. The number of corals in the CRO is variable along the generations, but since the number of function evaluations is fixed, the computational effort of the algorithm in the evaluation of new algorithms is similar. Crossover operator in the EA and broadcast spawning utilize the same operation, whereas mutation and brooding also resort to the same approach towards forming new individuals/corals. Therefore the main difference between these two approaches lies on the selection/larvae setting processes. The selection of the EA usually involves comparison between a fixed number of individuals (consider, e.g., a selection using ranking), whereas the larvae setting process is carried out until a free space or a worse coral is found or a maximum number of tries *κ* are reached. The selection of the positions in the reef where a larva can be set is driven uniformly at random. Thus, at the beginning of the CRO, the number of comparisons between corals is small (there are quite free spaces in the reef), and at the last stages of the algorithm the number of comparisons tends to be *κ* for each coral. In the case of the EA, the number of comparisons is kept similar all along the algorithm. This should mean a slightly better behavior in computation time of the CRO versus the EA. In spite of these differences and analysis, the main factor of computational complexity of these approaches is the number of function evaluations, and if this parameter is fixed, the differences in computation time between the different algorithms are negligible. This has been empirically checked in the experimental section of this paper, where all algorithms run within a very similar computation time.

## 4. Experiments and Numerical Results

In this paper we carry out a first performance assessment of the proposed CRO algorithm in different test problems. Specifically, different well-known continuous and discrete benchmark problems are under consideration: continuous analytical functions and several instances of the* Max Ones*,* 3-bit Deceptive,* and* MAX-3SAT* functions. Besides, the well-known traveling salesman problem (TSP) will be also included in our study. To end with, we finally show the performance of the CRO approach in two practical problem instances: optimum mobile network deployment and off-shore wind farm design.

We have selected other metaheuristic algorithms for comparison: evolutionary algorithms and genetic algorithms (EA and GA, [1]), harmony search (HS, [25]), particle swarm optimization (PSO, [7]), and differential evolution (DE, [4]), which have obtained excellent results in a wide range of optimization problems during the last years. Regarding the continuous benchmark problems, we have compared the results obtained by the CRO in the same problems tackled in [43], where different hybrid EAs are described, and also in different larger-dimensional problems described in [3]. On the other hand, in the case of the discrete benchmark problems we have assessed naïve versions of all the considered techniques. When specific operators must be included due to the intrinsic characteristics of the problem at hand (such as the TSP instances), such operators have been included in all the compared algorithms.

Following this rationale, the encoding strategy used to represent the produced solutions for the aforementioned problems is set identical for all the algorithms under comparison. Specifically, real encoding has been adopted for the continuous benchmark problems, whereas the* Max Ones*,* 3-bit Deceptive,* and* MAX-3SAT* problems resort to standard binary encoding, and the TSP utilizes permutations for representing a path among all cities. In the TSP we have used existing operators to manage crossover and mutation in permutation encoding [44–46]. On the other hand, values of all parameters controlling the CRO approach have been set to be comparable to that of its counterparts tested in every benchmark function. Therefore we have kept the number of function evaluations constant for all the compared algorithms in* Max Ones* (15000) and TSP (20000), whereas for the* 3-bit Deceptive* problem the total number of function evaluations is set to 50000 for GA and HS and 30000 for the proposed CRO. In the* MAX-3SAT* problem the number of function evaluations has been set to 15000 for all the algorithms. In the continuous benchmark functions, we have set the number of function evaluations to be comparable with the results in [43] (first set of functions), and we have set it to 10000 in the comparison with larger dimensional functions (CRO versus PSO, the best algorithms in the first set of functions). For every simulation instance 30 executions of each algorithm have been launched so as to obtain well-sampled performance statistics (best, average and standard deviation of the metric after all iterations are done). Note that the size of the population −*N* × *M* for CRO, population length *L* for the GA, and harmony memory size HM for HS have been set equal for all the experiments for the sake of fairness in the comparison of the algorithms: in the* Max-Ones* and* MAX-3SAT* problems *N* × *M* = 5 × 10, *L* = 50 and HM = 50, in the* 3-bit Deceptive* problem *N* × *M* = 10 × 10, *L* = 100 and HM = 100 and in the TSP *N* × *M* = 10 × 10, *L* = 100, and HM = 100. The CRO parameters *F*_*b*_ and *ρ* has been set to *F*_*b*_ = 0.9 and *ρ* = 0.7, unless otherwise stated in the discussion on the specific simulated application.

For the sake of validating the statistical significance of the obtained results, the distributions of the metric values obtained by the different algorithms on each scenario (groups) have been compared by means of a nonparametric Kruskal-Wallis test [47]. This test represents the nonparametric version of the classical one-way ANOVA and is an extension of the Wilcoxon rank sum test to groups larger than 2. To this end, the test compares the medians of the group, and returns the *P* value for the null hypothesis that all samples are drawn from the same population (or equivalently, from different populations with the same distribution). If the *P* value is lower than a predefined *α*, we can infer that the null hypothesis does not hold, that is, at least one sample median in the group is significantly different from the others, with (1 − *α*) level of confidence, then to determine which sample medians are statistically different, we have applied this multiple comparison procedure with *α* = 0.05 (thus, with a 95% level of confidence).

### 4.1. CRO Evaluation in Continuous Benchmark Problems

This first round of experiments includes four well-known benchmark functions, on which the proposed CRO is comparatively assessed with respect to different hybrid evolutionary algorithms described in [43]. In these experiments we have incorporated Gaussian and Cauchy mutations [3] in the internal reproduction (brooding) of the corals in order to accommodate the corresponding operator to the real encoding of the solutions. In the Gaussian mutation we have established a fixed standard deviation *σ* = (max⁡−min⁡)/100, where max⁡ and min⁡ are the maximum and minimum values that each component of the solution can take, whereas in the Cauchy mutation the value of the *τ* parameter has been fixed to 1 following the guidelines in [3]. The rest of operators in the CRO are the ones shown in Section 3. The first 4 rows of Table 1 summarize the details of the considered continuous benchmark functions.

Table 2 lists the results obtained by three different versions of the CRO (with Gaussian, Cauchy and Gaussian-Cauchy internal reproduction) in the benchmark functions tackled in this first round of experiments. We also include the results for different versions of the hybrid evolutionary algorithm proposed in [43], labelled as hybrid adaptive evolutionary algorithm (HAEA), and the results obtained with the PSO algorithm. It is straightforward to note that the CRO approach is able to obtain better results than the different versions of HAEA consistently, and with statistical significance positively checked through Kruskal-Wallis tests, in all the functions under consideration. The inclusion of both Gaussian and Cauchy mutations in the brooding coral reproduction (always maintaining the number of functions evaluations) appears to improve the performance of the CRO solver. Note that the PSO approach obtains results similar to the CRO, improving the best result obtained in some of the functions. In order to clarify the performance of the CRO versus the PSO, we have carried out some different tests of these algorithms in objective functions of larger dimensions, taken from [3] (functions *F*_1_ to *F*_7_ in Table 1). In this case the comparison of the proposed CRO versus the PSO algorithm is carried out with 1000 function evaluations per run.  Table 3 shows the obtained statistical performance metrics: the performance of both algorithms results to be quite similar (so dictates the statistical irrelevance by the Kruskal-Wallis test when applied on both result sets), though the CRO slightly, yet without statistical relevance, outperforms the PSO in 5 out of the 7 evaluated functions. This observation elucidates that the CRO algorithm renders a satisfactory performance level in continuous optimization problems.

### 4.2. CRO Evaluation in Discrete Benchmark Problems

The first discrete benchmark problem considered in this second stage is the well-known* Max Ones* problem, often used in a number of previous works aimed at evaluating different approaches of genetic algorithms (e.g., see [43, 48] and references therein). This optimization problem is defined in a binary search space *S* = {0,1}^*n*^, where *n* stands for the dimension of the space. The* One Max* problem is then defined as

(1) $$\begin{array}{c} \underset{x\in S}{\max}f\left(x\right)=\frac{100}{n}\overset{n}{\underset{i=1}{\sum }}x_{i}\left[\%\right]. \end{array}$$

Despite the evident simplicity of its definition, this problem is challenging for optimization algorithms when dealing with large values of the space dimensionality *n*.

Table 4 summarizes the results (maximum, average and standard deviation) obtained by CRO, GA, and HS in* Max Ones* instances of varying size from *n* = 50 to *n* = 500. As one may expect, in the scenarios of smallest dimension all the utilized heuristic approaches are able to obtain the optimum solution (100%) in every run of the algorithm. However, when the dimensions of the simulated problem increase, the differences between the CRO and the other tested algorithms become more significant. Specially remarkable is the fact that the CRO obtains the best value in all the instances with a very high probability (over 99% of the times in which the algorithm was run). HS also obtains good solutions, but notably worse than the GA even in the smallest instances. By contrast, the CRO clearly dominates GA and HS, specially in the largest* Max Ones* instances.

The second discrete benchmark problem addressed in this second phase is the maximization of the aforementioned* 3-bit Deceptive* function, which has been previously utilized to evaluate different improvements in genetic and evolutionary heuristics [43]. The 3-bit* Deceptive* function is a binary optimization problem defined in blocks of 3 bits. Each 3-bit block is assigned a value according to Table 5. The optimization of the function is known to be computationally hard for heuristic algorithms, since the 111 block (optimum since it is assigned the highest value) is “surrounded” by low-valued blocks of two 1s (i.e., with small Hamming distance with respect to 111). Different size functions (integer multiple of 3) are considered in this study; that is, *n* = {15,30,45,60,75,90,105,120}.

Table 6 shows the results obtained by the CRO in the considered 3-bit Deceptive functions, and its comparison to those of HS and GA. In this problem the CRO clearly obtains the best results among all the compared algorithms. Indeed, it is able to obtain the optimum (maximum) value in all the instances and in almost every executed run. The performance of the alternative algorithms degrades significantly in the largest instances, though in the smallest ones the GA is able to obtain the optimum value.

Finally, we have carried out a small test in several* MAX-3SAT* instances [49]. The* MAX-3SAT* is a well-known NP-complete optimization problem whose inherent complexity has motivated its wide adoption as a benchmark to assess the performance of different search algorithms. In this case five different* MAX-3SAT* instances of 20 clauses each have been considered, over which the performance of the CRO algorithm has been contrasted to that of HS and GA under the same operational setup (number of fitness evaluations per execution, solution encoding approach and parameter set optimized beforehand via intensive simulation). As Table 7 shows the results obtained. As can be seen, the CRO and GA are able to obtain the optimal result in all the considered instances, as opposed to the HS approach, which is not able to obtain the optimal result. Comparatively, both CRO and GA seem to perform similarly, as further supported by the lack of statistical significance of the results of both algorithms computed by the aforementioned Kruskal-Wallis test.

#### 4.2.1. Experiments in the Traveling Salesman Problem

The experimental discrete-variable benchmark follows by applying the proposed CRO algorithm to the TSP [45], which is a classical combinatorial optimization problem defined in the following way: given a finite number of cities along with the distance between each pair of them, the TSP consists of finding the shortest possible route visiting each city exactly once and returning to the origin city. Mathematically, let *V* denote the set of cities and *O* a Hamiltonian cycle (In graph theory, a Hamiltonian cycle is a cyclic path in an undirected graph that visits each vertex exactly once.) in *V*. Having these definitions in mind, the TSP hinges on finding the Hamiltonian cycle O* that minimizes the sum of the distances between all the cities visited in the order stated by O*, that is, that minimizes the objective function

(2) $$\begin{array}{c} f\left(O\right)=\left(\overset{|V|-1}{\underset{k=1}{\sum }}d\left(O\left(k\right),O\left(k+1\right)\right)\right)+d\left(O\left(\left|V\right|\right),O\left(1\right)\right), \end{array}$$

where |·| denotes cardinality, *O*(*k*) indicates the *k*th vertex (city) in the Hamiltonian cycle *O*, and *d*(*a*, *b*) stands for the distance measurement between city *a* and *b*.

In this paper we use different instances of the TSP with increasing number of cities. In a first round of experiments, we have set TSP instances of |*V*| = {30,40,50,75,100} cities, and generated 5 different TSP instances for each size. Hereby, we consider 25 different problems in this first analysis.  Table 8 collects the results (again, in best/average/standard deviation format) of CRO, GA, and HS when averaged over 30 runs of each algorithm. It is straightforward to conclude the CRO clearly outperforms statistically GA and HS in all the considered instances. To be concise, in the TSP instances with |*V*| = 30 nodes all the algorithms obtain the same minimum value; however, the average value over 30 runs is better for CRO. In the rest of TSP instances the CRO clearly outperforms GA and HS in all cases. Furthermore, the differences between the CRO and alternative metaheuristics become wider as the size of the TSP increases, as the computed statistics clearly show. Also remarkable is the fact that for all instances with |*V*| ∈ {50,75,100}, Kruskal-Wallis tests performed on the results of the compared metaheuristics confirm their statistical significance.

In order to further buttress this last observation, we have first carried out two extra experiments in very large TSP instances, that is, with |*V*| = {200,400}. The results of these experiments shown in Table 9 indicate that indeed the CRO performs remarkably better than its GA and HS counterparts, with statistical significance verified by Kruskal-Wallis. This set of TSP experiments concludes with a benchmark in a well-known TSP instance (“Berlin 52”), publicly available in the Internet.  Table 10 summarizes the results obtained by CRO, GA and HS in this problem, whereas Figure 4 shows the distribution of the cities in this problem, and the structure of the distance matrix, the best solution found by the CRO and the evolution of the best coral (solution) produced by the algorithm. Note that the CRO approach clearly obtains the best statistical results, again with proven statistical relevance by Kruskal-Wallis tests.

### 4.3. Experiments in a Practical Application Scenario: A Mobile Network Deployment Problem

In order to shed light on the performance of the CRO approach in a practical application, a mobile network deployment problem recently tackled in [50] has been chosen. Coined as the mobile network deployment problem (MNDP), it essentially consists of positioning a set of base transceiver stations (BTS) controllers taking into account a threefold criterion: maximization of the coverage, minimization of the deployment cost, and minimization of the electromagnetic pollution generated by newly allocated base stations controllers. A thorough statement of the problem can be found in the above reference [50]. The MNDP tackled in this study is located at Alcalá de Henares (Madrid, Spain), with specific details available in [50].  Figure 5 shows the location of the city under study, and the points considered where a BTS controller can be installed. The CRO approach has been compared to the evolutionary approach (EA) proposed in [50] that provided the best results so far in this problem. Both algorithms were run with the same solution encoding strategy, repairing heuristics and number of fitness evaluations.

Table 11 summarizes the results attained by the EA in [50] and the proposed CRO in this application scenario. As can be noticed from this table, CRO outperforms EA: although the solution produced by the CRO involves 12 BTS controllers versus 10 in the case of EA, it results in a lower cost. The noncoverage part of the objective function is also better in the case of the CRO solution, whereas the electromagnetic field is quite similar in both solutions.  Figure 6 shows the best solution found by the CRO and EA approaches, where the differences between the solutions found by the two approaches can be visually assessed.

### 4.4. Experiments in a Practical Application Scenario: Design of Off-Shore Wind Farms

The second practical application in which the proposed CRO is shown to yield an excellent statistical performance focuses on the optimal design of off-shore wind farms. In this setup the main objective is to maximize the production of the facility. Automatic wind farm design is indeed a hot topic in wind engineering [51]. Specifically, different computational optimization methods have been applied to the design of off-shore wind farms [52–55], most of them involving metaheuristic approaches, in particular evolutionary computation. In this section the optimal design of an off-shore wind farm is tackled by using the proposed CRO algorithm, an evolutionary algorithm (EA, [1]) and a differential evolution approach (DE, [4]). The specific problem is described in Figure 7, which shows the feasible points of turbine locations and their enveloping silhouette (with a uniform separation of 5 rotor diameters in order to reduce wake disturbances and effects) of an off-shore wind farm located at northern Europe. There are 73 possible locations for turbines in the considered wind farm, and the objective is to install 20 wind turbines in such a way that the production of the wind farm is maximized. We consider the* Bonus* 1.3 MW wind turbine model, and we resort to the Open Wind software ([56], freely available) for the corresponding wakes calculation and wind farm production estimation of the different layouts. All the compared algorithms utilize the same encoding approach, that is, integer numbers between 1 and the maximum number of feasible location sites in the wind farm. The EA includes a tournament selection, two-point crossover, and random mutation with a probability of 0.1. The chosen DE approach is a classical DE/rand/1/bin, with select weighting factor *F* = 0.8. Regarding the CRO approach, a 15 × 5 reef was considered, with an initial *ρ*_0_≃0.7 and parameter *F*_*b*_ = 0.9 (ninety percent of corals are considered as broadcast spawners). All the compared algorithms have been run until the number of objective function evaluations is 3000.

Table 12 compares the best solutions found by the three compared algorithms. Note that the CRO approach produces the layout with the best production, outperforming the EA and DE algorithms.  Figure 8 shows the best layout obtained by the CRO approach. Note that the wind turbines location tend to occupy the external upper zones of the wind farm. Since the wind rose in the zone of study has a predominant north-west component, the solution obtained is good, since the algorithm tries to locate the maximum number of turbines at the upper left-hand of the wind farm, so these turbines are not affected by wakes disturbances from other turbines.

## 5. Conclusions

In this paper we have presented a novel algorithm to solve optimization problems, inspired by the process of coral reefs formation and guided by coral reproduction, reef expansion, and fight for the space in the reef. The algorithm, named as the coral reef optimization (CRO) algorithm, is a kind of cellular evolutionary algorithm rendering very good properties of convergence to global optima. In this paper we have studied the main characteristics of the proposed CRO and analyzed its comparison to other existing metaheuristic approaches in different benchmark problems and two practical applications of mobile network deployment in Spain and the optimal design of an off-shore wind farm in northern Europe. The promising obtained results encourage the application of the proposed CRO approach to other practical optimization paradigms of high complexity.

## Figures and Tables

**Figure 1:** Illustrative recreation of a coral sexual reproduction by broadcast spawning: larvae are massively released into the water.

**Figure 2:** Coral reef simulation; (a) grid; (b) corals and holes in the reef.

**Figure 3:** Flow diagram of the proposed CRO algorithm.

**Figure 4:** TSP instance “Berlin 52” and solution by the proposed CRO algorithm.

**Figure 5:** City of the study (Alcalá de Henares, Madrid) and electromagnetic field measurement points; (a) situation of Alcalá de Henares, in Madrid, Spain; (b) electromagnetic field measurement points considered at Alcalá de Henares.

**Figure 6:** Best individual found by the CRO and EA algorithms in the MNDP considered at Alcalá de Henares; (a) CRO solution; (b) EA solution.

**Figure 7:** Off-shore wind farm considered and feasible locations to install wind turbines.

**Figure 8:** Best layout obtained by the CRO algorithm.

**Table 1:** Summary of the continuous benchmark functions considered in this paper.

Function	Expression	*n*	Feasible region
Rosenbrock	*f*_1_(*x*) = 100 · (*x*_1_^2^−*x*_2_)^2^ + (1−*x*_1_)^2^	2	[−2.048,2.048]^2^
Schwefel	$f_{2}\left(x\right)=418.9829\cdot n+\overset{n}{\underset{i=1}{\sum }}\left[-x_{i}\cdot \sin\left(\sqrt{\left|x_{i}\right|}\right)\right]$	10	[−512,512]^*n*^
Rastrigin	$f_{3}\left(x\right)=A\cdot n+\overset{n}{\underset{i=1}{\sum }}\left[x_{i}^{2}-A\cdot \cos\left(2\pi x_{i}\right)\right]$	10	[−5.12,5.12]^*n*^
Griewank	$f_{4}\left(x\right)=1+\overset{n}{\underset{i=1}{\sum }}\left[\frac{x_{i}^{2}}{4000}\right]-\prod_{i=1}^{n}\left[\cos\left(\frac{x_{i}}{\sqrt{i}}\right)\right]$	10	[−600,600]^*n*^
*F*_1_	$F_{1}=\overset{n}{\underset{i=1}{\sum }}x_{i}^{2}$	30	[−100,100]^*n*^
*F*_2_	$F_{2}=\overset{n}{\underset{i=1}{\sum }}\left|x_{i}\right|+\prod_{i=1}^{n}\left|x_{i}\right|$	30	[−10,10]^*n*^
*F*_3_	$F_{3}=\overset{n}{\underset{i=1}{\sum }}{\left(\overset{n}{\underset{i=1}{\sum }}x_{j}\right)}^{2}$	30	[−10,10]^*n*^
*F*_4_	*F*_4_ = max⁡_*i*_⁡(|*x*_*i*_ | , 1 ≤ *i* ≤ *n*)	30	[−100,100]^*n*^
*F*_5_	$F_{5}=\overset{n}{\underset{i=1}{\sum }}\left[100\cdot {\left(x_{i+1}^{2}-x_{i}\right)}^{2}+{\left(1-x_{i}\right)}^{2}\right]$	30	[−30,30]^*n*^
*F*_6_	$F_{6}=\overset{n}{\underset{i=1}{\sum }}\left(\left\lfloor x_{i}+0.5\right\rfloor \right)$	30	[−100,100]^*n*^
*F*_7_	$F_{7}=\overset{n}{\underset{i=1}{\sum }}ix_{i}^{4}+\text{random}\left[0,1\right)$	30	[−1.28,1.28]^*n*^

**Table 2:** Results (mean/standard deviation) obtained in the different continuous benchmark functions tested.

Algorithm	Rosenbrock	Schwefel	Rastrigin	Griewank
CRO (G)	0.00000709/0.000005	0.000132/0.00000207	0.007154/0.003039	0.223783/0.058051
CRO (C)	0.00000722/0.000006	0.000132/0.00000158	0.006713/0.002297	0.035024/0.019209
CRO (G + C)	0.00000229/0.000001	0.000131/0.00000145	0.004304/0.001564	0.053141/0.019543
HAEA (XUG)	0.000509/0.001013	0.005599/0.011702	0.053614/0.216808	0.054955/0.029924
HAEA (XU)	0.004167/0.004887	1.362088/0.932791	0.240079/0.155614	0.530857/0.227458
HAEA (XG)	0.001322/0.003630	140.5647/123.7203	7.731156/3.223595	0.050256/0.025888
HAEA (GU)	0.000160/0.000258	201.9162/81.28619	6.320374/1.462898	1.586373/0.383703
PSO	0.00000227/0.000002	0.000134/0.00000196	0.004719/0.002319	0.05018/0.01814

**Table 3:** Comparison of CRO (G + C) versus PSO in different benchmark functions from [3]. Average and standard deviation of the results of the 30 runs are shown.

Algorithm	PSO	CRO (G + C)
*F*_1_	1.24 · 10^−3^/3 · 10^−3^	1.30 · 10^−3^/2 · 10^−4^
*F*_2_	2.1 · 10^−3^/7 · 10^−4^	1.83 · 10^−3^/3 · 10^−4^
*F*_3_	2.6 · 10^3^/1 · 10^2^	2.0 · 10^3^/4 · 10^2^
*F*_4_	7.5/0.8	6.2/0.7
*F*_5_	1.7 · 10^3^/3 · 10^2^	1.6 · 10^3^/1.5 · 10^2^
*F*_6_	7.1 · 10^−3^/2 · 10^−4^	1 · 10^−3^/6 · 10^−4^
*F*_7_	0.02/1 · 10^−2^	0.02/0.9 · 10^−2^

**Table 4:** Results obtained by CRO, GA, and HS in * Max-Ones* problems of increasing size. The results are shown in best/average/standard deviation over 30 runs of the algorithms.

*n*	CRO	GA	HS
50	100/100/0	100/100/0	100/100/0
100	100/100/0	100/100/0	98/95.67/0.92
150	100/100/0	100/100/0	94.67/90.84/1.13
200	100/99.98/9.12 · 10^−4^	100/99.93/0.17	90/87.32/0.88
250	100/99.97/7.3 · 10^−4^	100/99.81/0.25	86.80/84.64/1.04
300	100/99.96 /8.45 · 10^−4^	100/99.61/0.39	83.67/82.0700/0.62
350	100/99.96/9.8 · 10^−4^	100/99.21/0.46	81.4300/80.03/0.71
400	100/99.95/7.3 · 10^−4^	99.50/98.67/0.58	79.50/78.45/1.04
450	100/99.93/0.13	99.55/98.11/0.67	78.67/76.97/0.99
500	100/99.92/0.1	98.60/97.04/0.75	78/75.99/0.69

**Table 5:** Value assignment in the considered * 3-bit Deceptive* function.

Groups of 3 bits	Value
$\begin{array}{ccc} 1 & 1 & 1 \end{array}$	80
$\begin{array}{ccc} 0 & 0 & 0 \end{array}$	70
$\begin{array}{ccc} 0 & 0 & 1 \end{array}$	50
$\begin{array}{ccc} 0 & 1 & 0 \end{array}$	49
$\begin{array}{ccc} 1 & 0 & 0 \end{array}$	30
$\begin{array}{ccc} 1 & 1 & 0 \end{array}$	3
$\begin{array}{ccc} 1 & 0 & 1 \end{array}$	2
$\begin{array}{ccc} 0 & 1 & 1 \end{array}$	1

**Table 6:** Results obtained by CRO, HS, and GA in the considered * 3-bit Deceptive* instances. The results are shown in best/average/standard deviation over 30 runs of the algorithms.

*n*	CRO	HS	GA	Upper bound
15	400/400/0	400/399.66/1.82	400/400/0	400
30	800/800/0	800/792/8.05	800/795/6.82	800
45	1200/1200/0	1190/1159/14.93	1200/1179.3/13.37	1200
60	1600/1600/0	1560/1517.3/21.96	1590/1562.70/18.74	1600
75	2000/2000/0	1910/1882/20.97	1990/1940.30/22.04	2000
90	2400/2400/0	2280/2243/22.63	2340/2297.30/21.16	2400
105	2800/2799.70/1.82	2660/2598.80/34.20	2730/2687.70/27.75	2800
120	3200/3200/0	2990/2924.8/37.90	3090/3049/21.22	3200

**Table 7:** Results obtained by CRO, HS, and GA in the considered * MAX-3SAT* instances (20 clauses). The results are shown in best/average/standard deviation over 30 runs of the algorithms.

Instance	CRO	HS	GA
1	0/1.4000/1.1425	1/6.6500/3.7314	0/0.1500/0.4894
2	0/1.3000/0.8645	2/6.5000/3.6921	0/0.1500/0.3663
3	0/1.9000/1.0208	1/6.5000/3.1871	0/0.3000/0.4702
4	0/1.4000/1.2732	1/5.5000/2.7625	0/0.0500/0.2236
5	0/1.3500/1.0894	1/6.1500/2.9249	0/0.1000/0.4472

**Table 8:** Results obtained by the CRO, HS, and GA in the considered TSP instances. The results are shown in best/average/standard deviation over 30 runs of the algorithms. I1 to I5 denote the index of the TSP instance for each value of |*V*|.

CRO	I1	I2	I3	I4	I5
30	44.48/44.93/0.59	46.50/46.70/0.58	47.67/48.73/1.32	47.36/47.69/0.74	45.86/46.40/0.53
40	50.99/52.47/0.79	48.04/48.96/1.14	54.86/55.93/1.02	47.81/48.15/0.77	49.16/50.25/1.00
50	59.47/62.02/1.75	54.51/56.34/1.63	57.73/58.97/1.34	58.14/60.16/1.09	57.92/59.77/1.19
75	75.48/78.41/1.61	72.16/75.07/1.98	77.53/81.16/2.04	75.40/80.49/2.17	72.04/6.28/0.05
100	108.03/111.98/2.78	108.26/115.38/3.40	106.93/113.81/3.81	109.35/115.38/2.75	107.79/113.81/3.02

GA	I1	I2	I3	I4	I5

30	44.48/45.68/1.26	46.50/47.02/1.19	47.67/49.20/1.20	47.36/48.30/1.42	45.86/47.05/0.88
40	51.60/53.86/1.31	48.12/51.15/1.68	55.94/57.39/1.19	48.49/50.11/1.25	49.29/51.68/1.60
50	64.70/68.01/2.22	57.04/61.63/2.59	61.55/65.07/2.12	60.97/64.45/2.45	61.15/64.86/2.08
75	88.12/94.47/3.6864	85.29/91.91/3.17	90.78/98.84/3.67	89.96/100.16/4.29	85.78/92.89/3.32
100	125.42/132.25/4.54	132.47/139.58/4.26	125.07/135.86/5.30	126.05/137.31/4.91	127.28/137.76/5.49

HS	I1	I2	I3	I4	I5

30	44.48/46.63/1.70	46.50/48.28/2.29	47.67/50.10/1.73	47.36/48.99/1.86	45.86/47.89/1.27
40	51.44/55.37/2.04	48.04/52.36/2.59	55.45/58.06/1.92	47.93/51.73/2.48	49.59/53.98/2.40
50	66.26/72.47/2.96	59.16/65.21/3.52	63.43/69.58/4.32	62.9215/68.89/3.33	62.37/69.05/3.47
75	98.34/108.36/6.41	85.70/105.76/8.81	94.98/113.17/7.77	100.26/113.85/6.22	91.45/106.42/6.45
100	127.85/152.37/10.48	148.39/164.16/9.25	142.38/163.93/10.00	144.57/164.13/9.44	146.70/162.67/8.46

**Table 9:** Results obtained by the CRO, HS, and GA in TSP instances of large size (|*V* | = {200,400}). The results are shown in best/average/standard deviation over 30 runs of the algorithms.

CRO	
200	133.98/138.18/2.58
400	407.84/424.76/8.00

GA	

200	194.02/205.19/4.05
400	495.21/514.62/10.61

HS	

200	233.58/266.16/17.03
400	618.85/674.18/22.02

**Table 10:** Results obtained by the CRO, HS, and GA algorithms in the TSP instance “Berlin 52.”

GA	HS	CRO
7758/7967/108	7688/7983/218	7542/7752/233

**Table 11:** Best values obtained in the MNDP problem considered at Alcalá de Henares, by the proposed CRO and an existing EA. EF stands for electric field and NC stands for noncoverage percentage.

Algorithm	Min. fitness	EF (mV/m)	Cost (K€)	NC (%)	Number of BTSs
EA in [50]	0.21554	3.16	2.4	2.75	10
CRO	0.1991	3.54	2.3	1.77	12

**Table 12:** Comparison of CRO, EA, and DE algorithms in the off-shore wind farm design problem.

Algorithm	Energy production (GWh)
CRO	84.352
EA	84.256
DE	84.292
